# Clinical Evaluation of FOXO1 as a Tumor Suppressor in Prostate Cancer

**DOI:** 10.1155/2021/8773423

**Published:** 2021-09-13

**Authors:** Ning Yang, Jiawen Wu, Tiancheng Zhang, Fan Yang, Jinyan Shao, Chang He, Liang Qin

**Affiliations:** ^1^Department of Urology, Minhang Hospital, Fudan University, 170 Xin-Song Road, Shanghai 201199, China; ^2^Medical College of Soochow University, Soochow University, 199 Renai Road, Suzhou 215123, China; ^3^Department of Emergency, Minhang Hospital, Fudan University, China

## Abstract

**Objective:**

Prostate cancer (PCa) is considered the most serious cancer in the world. Nevertheless, the accuracy of current biomarkers, such as pathological staging, Gleason's score, and serum prostate-specific antigen (PSA) levels, is limited. FOXO1 is a key downstream effector of PTEN and a tumor suppressor in PCA, which has been reported extensively. However, the clinical relevance of FOXO1 in PCa remains unclear.

**Methods:**

In this study, we first detected its expression in four public databases to explore the clinical role of FOXO1. Verification of the knockdown effect of FOXO1 siRNA was performed by real-time PCR analysis. Changes in cell viability were assessed using cell counting kit-8 (CCK-8) assays. In addition, we verified the effect of FOXO1 on the PCa cell cycle using a cell cycle assay.

**Results:**

Herein, we found that FOXO1 was significantly downregulated in PCa tissues and was significantly associated with Gleason's score, age, biochemical recurrence (BCR), and lymph node (LN) status, while FOXO1 expression was independent of pathological staging and preoperative PSA levels. The Kaplan-Meier survival analysis showed that PCA patients with high FOXO1 expression were less likely to develop BCR compared with patients with low FOXO1 expression. In terms of function, FOXO1 inhibition significantly promoted the proliferation and cell cycle progression of PCa cells.

**Conclusions:**

In summary, our study suggests that FOXO1 may be one of the prognostic factors that describe the risk of PCa for BCR. These results suggest that FOXO1 may be a therapeutic target for PCa.

## 1. Introduction

Prostate cancer (PCa) is a male malignancy that has been diagnosed with the highest frequency worldwide [1]. In China, PCa incidence is ranked the seventh, and among the leading causes of cancer-related deaths, PCa ranks the tenth [2]. At present, for localized PCa, the most common treatment belongs to radical prostatectomy (RP) [3]. Unfortunately, for a long term after RP, biochemical recurrence (BCR) has happened to approximately 25-60% of PCa patients [4, 5]. Gleason's score, pathological stage, and serum prostate-specific antigen (PSA) level are the main biomarkers of prostate cancer. However, the accuracy of these tests has limitations [6–8]. Thus, identifying new biomarkers for PCa is critical for assessing prostate cancer risk, recurrence, and prognosis clinically.

FOXO1, which belongs to the Forkhead box O (FOXO) proteins, is important in regulating a course of biological processes, containing glucose homeostasis, cell differentiation, cell proliferation, and DNA damage repair [9]. Increasing evidence has suggested that FOXO1 is a key downstream effector of PTEN [10] and in an array of human cancers which include prostate cancer [11–13], gastric cancer [14], and lung cancer [15], and it acts as the tumor suppressor. However, the clinical relevance of FOXO1 in PCa remains unclear.

This research employed public databases to explore FOXO1 expression in PCa tissues. Next, the relations of FOXO1 expression with varied clinical features of the PCa patients, which includes age, pathological stage, LN status, Gleason's score, preoperative PSA level and recurrence-free survival, were statistically evaluated based on the TCGA dataset. We also explored the functional roles of FOXO1 by knocking down its expression in PCa.

## 2. Materials and Methods

### 2.1. Data Sources

The microarray gene expression profiles used in this study were as follows: GSE38241 [16], GSE55945 [17], and GSE6919 [18].

The downloads of the miRNA-seq data and RNA-seq data of prostate cancer were provided by The Cancer Genome Atlas (TCGA, https://tcga-data.nci.nih.gov/tcga/) data portal. Clinical information of those cases was also collected, including gender, anatomic organ subdivision, location lung parenchyma, tumor status, AJCC tumor pathologic pT, AJCC node pathologic pN, AJCC pathologic tumor stage, AJCC metastasis pathologic pM, tobacco smoking history indicator, EGFR mutation status, EML4-ALK translocation status, new tumor event dx indicator, and vital status.

### 2.2. RNA Interference

The purchase of the special small interference RNAs (siRNAs) for human FOXO1 (siFOXO1-1461, 5′-CAATTCGTCATAATCTGTCCCTACA-3′; siFOXO1-1325, 5′-CAACCTTCTCTCATCACCAACATCA-3′; siFOXO1-1731, CAGAACGTCATGATGGGCCCTAATT) and nonspecific siRNA (5′-UAGCGACUAAACACAUCAA-3′) was achieved in GenePharma (Shanghai, China).

### 2.3. Cell Culture and Transfection

The American Type Culture Collection (Manassas, VA) provided the purchase of PC-3 and LNCaP cells, and their confirmation was accomplished by the short tandem repeat (STR) analysis. RPMI-1640 medium was used to culture cells which contain 100 U/ml penicillin, 10% fetal bovine serum (Hyclone, South Logan, UT), and 100 *μ*g/ml streptomycin, and in an environment of 37°C in 5% CO_2_, those cells were cultured. Lipofectamine 2000 (Life Technologies) was employed to help transfect those cells with siRNAs.

### 2.4. Real-Time RT-PCR

The extraction of total RNA was completed through the employment of the TRIzol Reagent (Invitrogen). The reversion of cDNA was completed through the performance of the PrimeScript RT Reagent Kit (TaKaRa, Tokyo, Japan). Based on the protocol of the manufacturers, the ABI Prism 7900 platform (Bio-Rad, Hercules, CA) and the SYBR Green Supermix were used to amplify cDNA samples. The calculation of the relative expression level compared with GAPDH levels was carried out by utilizing the 2^−ΔΔCt^ approach. The primer sequences that were used were as follows: FOXO1 (forward, 5′-TCGTCATAATCTGTCCCTACACA-3′ and reverse, 5′-CGGCTTCGGCTCTTAGCAAA-3′); GAPDH (forward, 5′-CTGGGCTACACTGAGCACC-3′ and reverse, 5′-AAGTGGTCGTTGAGGGCAATG-3′).

### 2.5. Cell Proliferation Assay

Changes in cell viability have been studied through the performance of CCK-8 assays. Five thousand transfected cancer cells were cultured in 96-well plates. 10 *μ*l CCK-8 (Dojindo, Kumamoto, Japan) has been employed to quantify the viability of the cells. After being incubated for two hours, cell viability in the 96-well plates were detected by employing a PowerWave XS Microplate Reader (BioTek, Winooski, VT, USA).

### 2.6. Cell Cycle Assay

After transfection for 48 h, the incubation of the cells continued for 15 minutes with PBS which contains 50 ng/ml propidium iodide (PI), 0.03% Triton X-100, and 100 ng/ml RNase A. Then, the FACSCanto Flow Cytometer (BD Biosciences, San Jose, USA, CA) was run to carry out the detection of those cells, and ModFit LT 3.0 software was utilized to analyze the cell cycle data.

### 2.7. Statistical Analysis

The data were shown as mean ± standard deviation (SD) of no less than 3 determinations. Kaplan-Meier's analysis was employed to appraise the correlation existing between FOXO1 and the prognosis of prostate cancer, as well as overall survival. All the tests were operated as being two-sided. It is statistically significant when *P* was lower than 0.05. The SPSS software was employed to conduct the statistical analysis.

## 3. Results

### 3.1. FOXO1 Was Downregulated in Prostate Cancer

To detect FOXO1's clinical features, this study first researched its expression in four databases (GSE38241, GSE55945, GSE6919, and TCGA). As shown in Figure 1, compared with adjacent prostate tissues, in human PCa tissues, the FOXO1 mRNA's expression levels were notably lower.

### 3.2. Decreased Expression of FOXO1 Correlated with the Aggressive Progression in PCa

Table 1 calculated the correlations between FOXO1 mRNA expression and varied features by using TCGA. The results made clear the correlation existing between the decreased expression of FOXO1 expression and age (*P* < 0.0047), BCR (*P* < 0.0277), Gleason's score (*P* ≤ 0.001), and LN status (*P* < 0.0324), whereas no relation was found to exist between FOXO1 expression and pathological stage (*P* = 0.2908) or preoperative PSA level (*P* = 0.0841) (all shown in Table 1).

### 3.3. Downregulation of FOXO1 Correlated with Poor Prognosis in PCa

As shown in Table 1, FOXO1 had a lower expression in patients who experienced BCR (*P* ≤ 0.001; Table 1). We fully studied the influence that the FOXO1 expression brought to prostate cancer patients. In Table 2, there was indication provided by the univariate Cox regression analysis that correlation existed between the higher Gleason score and the FOXO1 expression and a notably shorter biochemical recurrence-free survival (Figure 2(a)).

The Kaplan-Meier analysis elucidated that compared with FOXO1-high patients, there were lower 5-year BCR-free survival rates in patients with low FOXO1 (Figure 2(b)). In order to research the probability of BCR, we also combined the FOXO1 expression with the pathological stage. Compared with those that had FOXO1 negative expression, the positive FOXO1 staining had a notable probability of BCR among the subsets of GS ≤ 7 tumors and pT3/4 (Figures 2(c) and 2(d)). These findings indicated that high FOXO1 expression might be a notable prognostic indicator for PCa.

### 3.4. Knockdown of FOXO1 Promoted Prostate Cancer Proliferation

We next validated the functional roles of FOXO1 in PCa cell lines. FOXO1 siRNA was used to knock down its expression. Our results showed that three siRNAs against FOXO1 could significantly reduce FOXO1 mRNA expression compared to the negative control (Figures 3(a) and 3(c)).

We then researched FOXO1's function concerning cell proliferation in PC-3 and LNCaP cells by using the CCK-8 assay and found that knockdown of FOXO1 could significantly inhibit prostate cancer cell proliferation. (*P* < 0.001; Figures 3(b) and 3(d)). Provided that the cell growth could be revealed by the cell cycle data, we used flow cytometry to study FOXO1's function on the cell cycle profile of LNCaP (Figure 4(a)) and PC-3 (Figure 4(b)) cells. Cells' percentage in the G1 phase was amplified and that in the S phase (*P* < 0.001) was released by knocking down FOXO1 in LNCaP and PC-3 cells. These findings revealed that by strengthening cell cycle progression, FOXO1 promoted the PC-3 and LNCaP cells' proliferation and growth.

## 4. Discussion

PCa is serious cancer all over the world. However, the accuracy of current biomarkers, such as pathological stage, Gleason's score, and serum PSA level, has limitations. In this research, we have identified that FOXO1 was notably downregulated in PCa tissues and related to various PCa patients' clinical functions and poor survival outcomes. We have also found that the knockdown of FOXO1 dramatically promoted the proliferation and progression of PCa cells.

Growing evidence has shown that FOXO1 is downregulated in various human malignancies which include cervical cancer [19], breast cancer [20], and endometrioid endometrial cancer [21]. However, the clinical relevance of FOXO1 in PCa remains unclarified. This study researched FOXO1 expression in four publicly available databases and found that FOXO1 was notably downregulated in PCa samples. The correlation between the decreased expression of FOXO1 expression and BCR (*P* < 0.0277), Gleason's score (*P* ≤ 0.001), LN status (*P* < 0.0324), and age (*P* < 0.0047) (all shown in Table 1) has been demonstrated by TCGA data analysis. This analysis has also verified that FOXO1 expression was not pertinent to pathological stage (*P* = 0.2908) and preoperative PSA level (*P* = 0.0841) (all shown in Table 1). In the Kaplan-Meier outcomes, we have demonstrated that compared with FOXO1-low patients, PCa patients who had high FOXO1 expression had a low potential for obtaining BCR.

FOXO1, a key downstream effector of PTEN, is widely reported as a tumor suppressor in PCa. Other regulators in PCa, including AR pathways and miRNA, can also inhibit the expression of FOXO1. Huang et al. [22] showed that androgens negatively regulated FOXO1 expression through a proteolytic mechanism. Recently, reports also showed that a series of miRNAs, including miR-182 [13] and miR-96 [12], promoted PCa progression via inhibiting FOXO1 expression. In this research, we also evaluated the function of FOXO1 in PCa and found that the knockdown of FOXO1 dramatically propelled the LNCaP and PC-3 cells to proliferate and progress, and this accords with previous studies.

This study has some limitations. First, the mRNA and protein levels of FOXO1 need to be verified in clinical samples. Second, clinical samples should be collected to further explore the clinical value of FOXO1. In future studies, we will collect more prostate cancer patient samples to explore the correlation between FOXO1 expression and clinical parameters (including clinical stage, age, and survival time).

## 5. Conclusions

In conclusion, our study has shown that FOXO1 might be a prognostic factor in the prediction of BCR's risk for PCa. Furthermore, the proliferation and progression of PCa were promoted significantly by the knockdown of FOXO1. These results indicate the potential of FOXO1 being a target of PCa treatment.

## Figures and Tables

**Figure 1:** FOXO1 was downregulated in prostate cancer. The comparison between FOXO1 expression levels in normal prostate tissues and prostate tumors is shown in four gene expression data, namely, GSE38241 (a), GSE55945 (b), GSE6919 (c) and TCGA (d), which are all publicly available Significance holds if *P* is below 0.05 (^∗^*P* < 0.05; ^∗∗^*P* < 0.01; ^∗∗∗^*P* < 0.001).

**Figure 2:** The Kaplan-Meier curve analyses of biochemical recurrence-free survival of prostate cancer patients. Comparison between FOXO1 expression levels in Gleason score (6 + 7) prostate tumors and Gleason score (8 + 9) prostate tumors in TCGA is shown in (a). Based on the expression of FOXO1, that of FOXO1 and Gleason score, and that of FOXO1 and tumor pT (b–d), respectively, provide the Kaplan-Meier curves for biochemical recurrence-free survival in patients who had prostate cancer. Significance holds if *P* is lower than 0.05 (^∗^*P* < 0.05; ^∗∗^*P* < 0.01; ^∗∗∗^*P* < 0.001).

**Figure 3:** Cell proliferation in PCa cells promoted by the knockdown of FOXO1. (a, c) Expression of FOXO1 mRNA after being transfected with the indicated siRNAs in LNCaP and PC-3cells. (b, d) Cell proliferation in LNCaP (b) and PC-3 (d) cells promoted by the knockdown of FOXO1. Each of the experiments was conducted in triplicate (*n* = 3). Data were recorded as the mean ± SD (^∗∗^*P* < 0.01; ^∗∗∗^*P* < 0.001; Student's *t*-test).

**Figure 4:** Cell cycle in PCa cells promoted by the knockdown of FOXO1. In LNCaP (a) and PC-3 (b) cells, cells' percentage in the G1 phase was decreased and that in the S phase was increased by the knockdown of FOXO1. Significance holds if *P* is below 0.05 (^∗^*P* < 0.05; ^∗∗^*P* < 0.01; ^∗∗∗^*P* < 0.001).

**Table 1:** Correlation between FOXO1 expression and clinicopathologic features in PCa patients.

Features	Number	FOXO1 expression		*P* value
		Low	High	
Age (*n* = 380)				
<60	183	88	95	0.0362
>60	197			
Pathological stage (pT) (*n* = 378)				
pT2a-pT2c	157	72	85	0.2908
pT3a-pT4	221	118	103	
Lymph node status (*n* = 312)^∗∗^				
Positive	51	32	19	0.0032
Negative	261	121	140	
Preoperation PSA level (ng/ml) (*n* = 338) Median (range)		11.81 ± 1.008	9.612 ± 0.7684	0.0841
Gleason score (*n* = 380) ^∗∗^				
Gleason ≤ 7	243	100	123	0.0057
Gleason ≥ 8	137	70	47	
Biochemical recurrence(*n* = 315) ^∗∗^				
Yes	34	24	10	0.0016
No	281	131	150	

^∗^*P* < 0.05, ^∗∗^*P* < 0.01, ^∗∗∗^*P* < 0.001.

**Table 2:** Multivariate analysis of BCR-free survival for all PCa patients.

Comparison	*P* value	Hazard ratio for recurrence	95% CI
Lymph node status	0.904	0.939	0.335, 2.629
FOXO1 expression	0.027	1.390	0.675, 4.095
Gleason score	0.056	0.361	0.122, 1.068
Pathological stage	0.073	0.278	0.059, 1.298
Age	0.806	0.895	0.368, 2.174
Preoperation PSA	0.376	0.644	0.244, 1.704

## Data Availability

All data analyzed during this study were obtained from the published article or are available from the corresponding authors on reasonable request.
